RETRACTED

# The Effect of Hyperlipidemia on Peri-implant Health: A Clinical and Radiographical Prospective Study

**DOI:** 10.1155/2023/7570587

**Published:** 2023-04-26

**Authors:** Paolo De Angelis, Edoardo Rella, Paolo Francesco Manicone, Giulio Gasparini, Valerio Giovannini, Margherita Giorgia Liguori, Francesca Camodeca, Giuseppe De Rosa, Camilla Cavalcanti, Antonio D'Addona

**Affiliations:** ^1^Department of Head and Neck and Sensory Organs, Division of Oral Surgery and Implantology, Fondazione Policlinico Universitario A. Gemelli IRCCS–Università Cattolica del Sacro Cuore, Rome, Italy; ^2^Department of Head and Neck and Sensory Organs, Division of Oral and Maxillofacial Surgery, Fondazione Policlinico Universitario A. Gemelli IRCCS–Università Cattolica del Sacro Cuore, Rome, Italy

## Abstract

High levels of cholesterol and triglycerides may have a negative effect on the immune system and bone health, leading to lower bone mineral density, an increased risk of osteoporosis, and bone fractures, and could therefore also be related to a significant worsening of peri-implant health. The purpose of the following study was to evaluate whether the altered lipid profile in patients who undergo implant insertion surgery represents a prognostic factor capable of influencing clinical outcomes. This prospective observational study was conducted on 93 subjects; patients were required to have taken blood tests to obtain triglycerides (TG), total cholesterol, low-density lipoprotein (LDL), and high-density lipoprotein (HDL) levels prior to the surgical procedure to classify them according to current American Heart Association guidelines. The outcomes considered were marginal bone loss (MBL) 3 years after implant placement, full-mouth plaque score (FMPS), and full-mouth bleeding score (FMBS) 3 years after surgery. A statistically significant correlation was found between hypertriglyceridemia and MBL as well as between total cholesterol and MBL. There is no statistically significant correlation between the variables analyzed and the secondary outcomes 3 years after implant placement. Peri-implant marginal bone loss may be influenced by hyperlipidemia. However, further studies are needed, with larger samples and more extensive follow-ups, to confirm these results.

## 1. Introduction

The atherogenic, or high-fat (HF), diet induces hyperlipidemia, a state with an abnormal lipid profile characterized by elevated blood concentrations of triglycerides, high levels of total and low density lipoprotein (LDL) cholesterol, and reduced levels of high density lipoprotein (HDL) cholesterol [1].

An HF diet is associated with the pathophysiology of several diseases, including atherosclerosis, vascular calcifications, and osteoporosis, which are major causes of morbidity and mortality in the aging population [2–5].

RETRACTED

The current American Heart Association guidelines define hyperlipidemia by levels of total cholesterol (>240 mg/dL), LDL cholesterol (>160 mg/dL), or triglycerides (>200 mg/dL). Because low HDL levels (<40 mg/dL in men and <50 mg/dL in women) are also considered atherogenic, the terms “dyslipidemia” and “atherogenic lipid profile” are also used [6].

Under conditions of hyperlipidemia, protein-bound lipid particles pass through the endothelial wall to the subendothelial level, where they are captured and oxidatively modified by reactive oxygen species produced by metabolically active nearby smooth muscle cells and macrophages. A similar phenomenon occurs in human osteoporotic bone, with lipid particles bound to oxidized proteins collecting at the perivascular and subendothelial levels. Osteoblasts can also oxidatively modify protein-bound lipid particles, and oxidized lipid products have been detected in the bone marrow of hyperlipidemic mice [7, 8].

Krieger et al. [9] showed an increase in the number of osteoclasts, inhibition of osteoblastic activity, and a reduction in bone remodeling in hyperlipidemic rats. According to Luegmary et al. [10], high-cholesterol levels can lead to an imbalance in the bone remodeling processes, reducing bone mass by increasing osteoclast activity and differentiation.

Because of the deleterious effects of hyperlipidemia on bone, it has been hypothesized that hyperlipidemia may interfere with bone grafting and dental implant therapy, as the quantity, quality, and healing potential of the host play an important role in the osseointegration and bone regeneration process [11–14].

Only one study investigated the effects of hyperlipidemia on implant osseointegration in mice by implant push-in test and microcomputed tomography (micro-CT) analysis. In this study, Keuroghlian et al. [15] found that mice fed a high-fat diet had a significantly increased chance of implant failure as well as reduced bone-implant interface formation and strength.

Three studies by the same author investigated the relationship between hypercholesterolemia and dental implant failure in humans, but none of the three reported any causal relationship between hypercholesterolemia and implant failure rates [16–18].

To the best of our knowledge, peri-implant tissue healing and bone graft maturation in the presence of hyperlipidemia have not yet been extensively studied.

The increasing number of patients with hyperlipidemia represents a challenge due to the high number of procedures and the risks of directly compromising clinical outcomes and increasing therapeutic failures.

RETRACTED

The present prospective study is aimed at testing the null hypothesis that hyperlipidemia does not influence peri-implant marginal bone level (MBL) 3 years after implant placement.

## 2. Materials and Methods

This prospective study enrolled 93 patients treated at the Department of Oral Surgery and Implantology of the Catholic University of the Sacred Heart of Rome. All investigations have been performed in accordance with the 1975 Declaration of Helsinki, revised in 2013 for ethical approval. All participants have provided written informed consent after receiving all relevant information regarding the objectives and procedures of the study.

Ethical approval was obtained from the Catholic University of the Sacred Heart, Rome, Italy (ID: 4130).

All surgeries were performed by the same trained and experienced surgeon.

Patients were selected on the basis of the following inclusion criteria:

1. Patients who needed a single implant to treat a partial edentulism
2. Healthy patient or stable periodontitis patient
3. Total cholesterol, LDL-cholesterol (LDL-c), HDL-cholesterol (HDL-c), and triglyceride values recorded no more than 3 months before enrollment
4. Age > 20 years

The exclusion criteria were as follows:

1. Periodontal disease
2. Taking any medication known to affect oral status and bone turnover or that contraindicate surgical treatments (therapy with immunosuppressants, corticosteroids, or bisphosphonates)
3. Previous radiotherapy or chemotherapy
4. Smokers
5. Excessive alcohol consumption
6. Conditions associated with an altered relationship between glycated hemoglobin and blood glucose such as sickle cell anemia, pregnancy, glucose-6-phosphate dehydrogenase deficiency, HIV, hemodialysis, recent transfusion, or erythropoietin therapy

The following factors were evaluated and collected prior to implant placement:

1. Age
2. Gender
3. BMI (Body Mass Index)
4. Ethnicity
5. Regenerative bone graft therapy prior to implant placement (yes/no)

Patients were classified according to the current American Heart Association guidelines [19].

Patients were divided into four groups based on triglyceride levels (1: <150 mg/dL, 2: 150–199 mg/dL, 3: 200–499 mg/dL, and 4: ≥500 mg/dL); into two groups based on total cholesterol levels (1: <200 mg/dL, 2: ≥200 mg/dL); into two groups based on LDL levels (1: <100 mg/dL, 2: ≥100 mg/dL); and into two groups based on HDL levels (women—1: ≥50 mg/dL, 2: <50 mg/dL; men—1: ≥40 mg/dL, 2: <40 mg/dL).

The following clinical outcome variables were assessed before surgery by the same operator, using a University of North Carolina periodontal probe (UNC15, Hu-Friedy, USA).

- Probing pocket depth (PPD)
- Full-mouth bleeding score (FMBS)
- Full-mouth plaque score (FMPS)

PPD was measured for each site and then averaged.

RETRACTED

Each patient underwent a preoperative cone-beam computed tomography (CBCT) scan to complete the preoperative planning and evaluate the bone volume. Before the surgical phase, all subjects were enrolled in a rigorous oral hygiene regimen.

Surgery was performed under local anesthesia (articaine 4% with epinephrine 1 : 100000). A crestal incision was performed, and it was continued intrasulcularly involving the mesial and distal tooth. A mucoperiosteal flap was raised, and the bone was exposed and carefully curetted. An osteotomic site was created following company protocol, and a bone-level implant was placed, with the implant neck positioned crestally. During the implant placement, primary stability was assessed via the insertion torque and hand testing; single sutures were placed to obtain a primary intention closure.

Patients were instructed to rinse twice daily with a 0.2% chlorhexidine mouth rinse. In addition, analgesics (Ketoprofen) were prescribed for the next 3 days according to individual needs. Patients were also instructed to refrain from mechanical plaque removal in the surgical site. The sutures were removed 7–10 days after surgery.

Four months after implant positioning, a digital or a conventional impression was taken. After prosthesis delivery, all the patients were enrolled in a periodontal maintenance program.

A CBCT scan was then taken at the 3-year follow-up.

The primary outcome of the study was the change in peri-implant MBL 3 years after implant placement, measured using the CBCT scan (Orthophos XG 3D, Sirona Dental Systems GmbH). The CBCT scan was transferred into a dedicated software system (Implant Studio, 3Shape, Copenhagen K Denmark) used to perform the measurements, carried out by one designated examiner. For the most accurate details, the study used a field of view of 5 × 5 cm with a voxel size of 100 *μ*m. All radiographic and tomographic images were taken by the same trained operator. On the CBCT coronal and sagittal section, the distances between the implant neck and the buccal/palatal bone and from the implant neck to the mesial and distal bone were measured in millimeters, and the higher value was considered for each implant.

Adverse events (e.g., wound infection, graft exposure, and soft tissue dehiscence or necrosis) were recorded during follow-up.

A sample size of 82 subjects was required to achieve a power of 80%, at a significance level of 0.05, expecting to build a final model with eight predictors with an effect size of 0.2.

### 2.1. Statistical Analysis

Categorical data were analyzed as absolute and relative frequency, whereas numerical data were reported as means and standard deviations.

RETRACTED

A multiple regression analysis was performed to evaluate the effects of the variables on MBL and FMBS; only the variables that had a statistically significant outcome in univariable models were inserted in the multivariable analysis. Statistical analysis was conducted using STATA (StataCorp. 2021. Stata Statistical Software: Release 17. College Station, TX: StataCorp LLC).

## 3. Results

The analyzed sample is composed of 93 patients, with a mean age of 56.97 ± 13.76. Tables 1–3 show the demographic, distribution, and periodontal data. All patients underwent the described implant surgery procedures; five patients were affected by postoperative complications.

The results of the univariable analysis are reported in Tables 4 and 5. A previous regenerative therapy, the occurrence of complications, higher BMI level, higher levels of triglycerides, higher levels of LDL cholesterol and total cholesterol, lower levels of HDL cholesterol, and a higher FMPS had an impact on the amount of MBL, according to the univariable model.

Only the variables that had a significant effect were inserted in the multivariable analysis, and the results are reported in Tables 6 and 7.

Only a previous regenerative therapy, a higher FMPS and higher levels of triglycerides and total cholesterol had an impact on the amount of MBL, according to the multivariable model. HDL and LDL had no effect in this model, even if patients who had a higher level of LDL and lower level of HDL revealed a notable increase in the MBL (Figures 1 and 2); this was probably caused by the high collinearity found in the present data sample because patients who had higher levels of cholesterol and triglycerides also had high levels of LDL and lower levels of HDL.

Regarding the FMBS, a significant effect was found only for the FMPS, according to the multivariable model.

## 4. Discussion

Implant therapy has become a widely used procedure for dental rehabilitation; it is considered safe and has a high survival and success rate, although certain conditions can affect the predictability of outcomes. One of these conditions may be an abnormal lipid profile due to its influence on the peri-implant hard and soft tissues [20].

The primary purpose of this study was to examine the hyperlipidemia influence on peri-implant marginal bone level (MBL) at 3 years after implant placement. Marginal bone loss surrounding dental implants is one parameter that has been commonly used to determine implant success and health and is associated with the long-term success of implant treatment [21]. Although bone regeneration is an efficient process in physiological conditions, many variables such as phlogosis, hormonal changes, and elevated serum lipid levels may be associated with the impaired or delayed healing process [22]. Recently, a correlation between atherosclerotic vascular disease and bone loss has been demonstrated [23], and it is accepted that a high-fat diet (HFD) reduces bone density and increases bone resorption activity [24]. The role of lipid and lipid-bound protein oxidation in the pathophysiology of osteoporosis has been reported by a variety of studies [25, 26].

RETRACTED

In their experimental study, Lu et al. [27] reported that the bone mineral content and the area of trabecular bone were significantly decreased in the HFD group compared to the controls. Moreover, they reported that in a cell culture study on aspirated bone marrow derived from mice, the colony-forming unit osteoblasts were significantly decreased in the HFD sample compared to the control [27].

The deleterious effects of HFD on osseointegration and stability of peri-implant hard tissues can be explained by more than one mechanism. At a cellular level, hyperlipidemic conditions lead to inhibition of osteogenic signaling, reductions in the number of mature osteoblasts, a higher expression of molecular markers of bone remodeling, enhancement of osteoclast differentiation and activity, and increased bone resorption [28, 29].

In clinical practice, the influence that the lipid profile can have on the peri-implant bone remains a subject of controversy. Some studies report a correlation between lipid levels and peri-implant bone; other studies conflict with these conclusions. The latter category includes a study by Dundar et al. [8] who reported no differences in bone-to-implant contact (BIC) 12 weeks after implant placement between rabbits following a 3-month high-fat diet versus normal diet.

Other authors have investigated the influence of the lipid profile on periodontal disease and alveolar bone resorption. Hyperlipidemia seems to have a dysregulatory effect on immune system and wound healing, increasing the susceptibility to periodontal disease and other infections [26, 30, 31].

Macri et al. [32] focused on the effect of an atherogenic cholesterol-rich diet on the alveolar bone loss in rats with ligature-induced experimental periodontitis, and they concluded that an atherogenic cholesterol-rich diet induced hyperlipidemia and appeared to be a risk factor for the onset and progression of experimentally induced periodontitis. However, Valera-Lopez's study on rabbits showed that HFD could exacerbate some aspects of periodontitis, but the presence of some oral microorganisms in the subgingival plaque is essential for this exacerbation [33]. Another study by Kırzıoğlu et al. [34] showed that no additive effect of cholesterol-enriched diet to alveolar bone loss (ABL) was found in rats with ligature-induced experimental periodontitis. The relationship between hyperlipidemia and periodontal disease may involve also the bacterial interaction. Choi et al., in a human study, performed a multivariable analysis and after adjusting for periodontitis and other potential risk factors found that a higher burden of periodontal bacteria was independently associated with lower HDL and higher TG in serum. This result may suggest also a possible link between exposure to periodontal bacteria and increased risk of dyslipidemia [19].

RETRACTED

It must be considered that most of the studies in the literature on this topic have been conducted using experimental animal models; therefore, one of the notable features of the present study consists in having taken a human experimental model as a reference.

The results of the present study demonstrate that the variables that appear to have the greatest effect on MBL are having received previous regenerative therapy, a higher FMPS, and higher levels of triglycerides and total cholesterol. At the same time, it seems that the levels of LDL and HDL do not have a statistically significant effect on the primary outcome. This was probably caused by the high collinearity found in the data sample.

The absence of correlation with LDL and HDL levels is in line with the results obtained from three studies by Alsaadi et al. conducted between [16–18]. In those three studies conducted on a human experimental model, the authors did not report any causal relationship between hypercholesterolemia and implant failure, but hypercholesterolemia was analyzed in association with many other local and systemic factors; consequently, the results may not be accurate. Furthermore, the method of measuring hypercholesterolemia had not been adequately clarified. Another retrospective cohort study did not find a significant association between an elevated triglyceride level and implant failure [23]. However, in the present study, MBL was analyzed as a primary outcome. Interestingly, in studies showing an inverse association between cholesterol levels and bone mineral density, this association is the same for both TG and LDL-cholesterol levels, whereas in our study, it was not the same [35, 36]. Therefore, further studies are required to better investigate the association between hypercholesterolemia and hypertriglyceridemia and their effect on bone metabolism.

Several in vivo animal studies demonstrate that a hyperlipidemic diet significantly increases implant loss as well as reduced bone-implant interface formation and strength. Obviously, human clinical correlation is required.

RETRACTED

The limitations of the present study are related to the lack of previous clinical studies analyzing the effect of hyperlipidemia on MBL, the small study sample, the relatively short follow-up, and the lack of a bacterial analysis. Furthermore, patients' lipid profile was measured only once, at the beginning of the study, and it could have suffered variations during the follow-up.

## 5. Conclusions

Despite the limitations of the present study, the results support the hypothesis that peri-implant marginal bone loss may be influenced by a condition of hyperlipidemia. However, further studies are needed, with a larger sample and more extensive follow-up, to confirm these results.

## Figures and Tables

**Figure 1:** Box plot outlining marginal bone loss distribution considering the LDL levels.

**Figure 2:** Box plot outlining marginal bone loss distribution considering the HDL levels.

**Table 1:** The demographic characteristics of the sample.

Variable	Absolute frequency
*Gender*	
Male	54
Female	39
*Race*	
Caucasian	87
Asian	3
Latino-American	2
Afro-American	1
*Previous regenerative therapy*	
Underwent a regenerative surgery	17
Did not undergo a regenerative surgery	76
*Adherence to the maintenance program*	
Followed the maintenance program	70
Did not follow the maintenance program	23
*Occurrence of complication*	
Suffered a complication	5
Did not suffer a complication	88

**Table 2:** The “nutritional” values of the sample.

Variable	Absolute frequency
*BMI*	
1	38
2	35
3	17
4	3
*Triglyceride levels*	
1	42
2	29
3	22
*Cholesterol levels*	
1	38
2	55
*LDL levels*	
1	42
2	51
*HDL levels*	
1	35
2	58

**Table 3:** The periodontal values of the sample.

Variable	Mean	Standard deviation
FMBS	15.48	4.40
FMPS	16.84	4.56
PPD	2.92	0.57
MBL	0.53	0.42

**Table 4:** The results of the univariable analyses for the outcome MBL.

Variable (MBL)	Coefficient	*P* value
Gender	-0.11	0.27
Age	0.005	0.16
Ethnicity	-0.37	0.70
Previous regenerative therapy	0.27	0.03^∗^
Adherence to the maintenance program	-0.39	0.7
Occurrence of complication	0.62	0.004^∗^
BMI	0.25	0.0001^∗^
Triglyceride levels	0.25	0.0001^∗^
Cholesterol levels	0.36	0.0001^∗^
HDL levels	0.31	0.002^∗^
LDL levels	0.29	0.003^∗^
FMPS	0.05	0.0001^∗^
PPD	0.13	0.13

**Table 5:** The results of the univariable analyses for the outcome FMBS.

Variable (FMBS)	Coefficient	*P* value
Gender	-0.87	0.34
Age	-0.01	0.75
Ethnicity	-0.3	0.70
Previous regenerative therapy	-0.8	0.94
Adherence to the maintenance program	-1	0.3
Development of complication	4.13	0.04^∗^
BMI	1.3	0.01^∗^
Triglyceride levels	0.6	0.27
Cholesterol levels	1.5	0.09
HDL levels	1.82	0.05
LDL levels	1.53	0.09
FMPS	0.57	0.0001^∗^
PPD	1.42	0.07

RETRACTED

**Table 6:** The results of the multivariable analysis for the outcome MBL.

Variable (MBL)	Coefficient	Confidence interval	*P* value
Previous regenerative therapy	0.23	0.03–0.44	0.02^∗^
Development of complication	0.15	-0.22–0.52	0.42
*BMI*			
2	0.05	-0.11–0.22	0.52
3	0.19	-0.05–0.44	0.12
4	0.66	0.24–1.09	0.003
*Triglyceride levels*			
2	0.17	-0.26–0.36	0.09
3	0.26	0.01–0.51	0.04^∗^
*Cholesterol levels*			
2	0.16	-0.21–0.54	0.4^∗^
*HDL levels*			
2	-0.10	-0.44–0.23	0.54
*LDL levels*			
2	-0.05	-0.27–0.17	0.66
FMPS	0.045	0.03–0.06	0.001^∗^

**Table 7:** The results of the multivariable analysis for the outcome FMBS.

Variable (FMBS)	Coefficient	Confidence interval	*P* value
Development of complication	2.49	-1.26–6	0.16
*BMI*			
2	1.05	-.61–2.7	0.52
3	0.64	-1.6–2.89	0.57
4	1.77	-2.47–6	0.4
FMPS	5	0.37–0.7	0.001

## Data Availability

The datasets used and/or analyzed during the current study are available from the corresponding author on reasonable request.
